The article "Consistency Analysis of CTLM Imaging and Mammography in the Diagnosis of Breast Tumor Lesions" was retracted in 2023. Reasons: signs of a paper mill; suspected computer-generated content; unreliable results or conclusions; lack of ethics approval or compliance.

# Consistency Analysis of CTLM Imaging and Mammography in the Diagnosis of Breast Tumor Lesions

**DOI:** 10.1155/2022/5391636

**Published:** 2022-03-29

**Authors:** Zhangjun Song, Huxia Wang, Xiaorui Feng, Xiaomin Yang, Pihua Han, Jing Zhao

**Affiliations:** ^1^Department of Oncology, Shaanxi Provincial People′s Hospital, Xi′an 710068, China; ^2^Department of Breast, Shaanxi Provincial Cancer Hospital, Xi′an 710061, China; ^3^Department of Radiation Oncology, Xi′an High-tech Hospital, Xi′an 710000, China

## Abstract

Objective. To analyze the consistency of preoperative CTLM imaging in the diagnosis of breast cancer lesions and postoperative pathological examination. Methods. The clinical data of 225 patients with breast tumor in our breast surgery department were collected. All patients underwent mammography, CTLM, and pathological examination. To analyze the image characteristics of breast CTLM imaging, calculate the diagnostic efficacy of CTLM imaging for breast tumors, and compare the image characteristics of CTLM imaging for benign and malignant tumors. Results. (1) Postoperative pathological examination showed that 136 cases (60.44%) of lesions were benign tumors, and 89 cases (39.56%) were malignant tumors. (2) The “spokes distribution” of normal breast CTLM images was interrupted. In the 3D reconstructed images, the morphology of the abnormal angiogenesis area is mostly irregular nonbanded structure, which is manifested as slab structure, spindle structure, spherical structure, diverticulum structure, inverted conical structure, rings structure, branched structure, and dumbbell structure. (3) The detection rate of breast tumor by CTLM imaging was 84.44%. The specificity and coincidence rate of CTLM imaging were higher than that of mammography (*P* < 0.05). (4) The features of CTLM imaging images of breast malignant tumors are mostly bright white locally, with irregular edges and obvious attenuation of laser signal, and the reconstructed shape of 3D images is mostly like a slab structure. Conclusion. CTLM imaging can provide related information of neovascularization in breast cancer lesions, which is basically consistent with pathologically confirmed lesions.

## 1. Introduction

According to the global cancer incidence and death rates released by the International Agency for Research on *Cancer* in 2020 [1], female breast cancer has surpassed lung cancer as the most common cancer. Factors such as women′s age [2], fertility [3], hormone use [4], and family history of breast cancer [5] affect the incidence of breast cancer. For example, the incidence of breast cancer increases with age. Annual physical examination is recommended for women younger than 40 years of age and can help patients screen for abnormalities early in the disease [6]. Physical examination of the breast usually involves routine imaging examinations, such as mammography [7]. There are some limitations to this examination. Breast density affects the rate of disease detection. For women between 40 and 79 years with fatty breasts, the sensitivity is 80–87%. However, for women with dense breasts, the sensitivity of the examination is significantly decreased [8]. Early detection of breast cancer lesions and accurate measurement of tumor size in abnormal lesions can help to develop accurate treatment protocols and improve patient prognosis. Radiologists are often unable to make an accurate diagnosis with only the results of routine imaging tests. Computed tomographic laser mammography (CTLM) is an optical imaging method [9]. The near-infrared laser with a wavelength of 808 nm can be used as the laser source, the oxygenated hemoglobin in the blood vessels of patients can be used as the natural contrast agent of human body, and the stimulated light can be absorbed and scattered [10]. Finally, abnormal vascular information was obtained by 3D image reconstruction. Abnormal angiogenesis plays a key role in tumor growth, nourishing the lesion and promoting the proliferation and migration of abnormal cells. In the examination of breast cancer, monitoring abnormal angiogenesis is of great significance. Therefore, 225 patients with breast tumors in this study were examined by routine mammography, CTLM imaging, and pathological examination, with mammography as the contrast, aiming to analyze the image characteristics of breast tumor measured by CTLM imaging and the consistency between the diagnosis of lesions and postoperative pathological examination.

The article "Consistency Analysis of CTLM Imaging and Mammography in the Diagnosis of Breast Tumor Lesions" was retracted in 2023. Reasons: signs of a paper mill; suspected computer-generated content; unreliable results or conclusions; lack of ethics approval or compliance.

## 2. Materials and Methods

### 2.1. General Data

A retrospective analysis was performed on breast tumor patients admitted to the Mammary Department of Shaanxi Provincial *Cancer* Hospital from January 2018 to February 2020. All patients were examined by mammography and CTLM. The treatment was operation, and the diagnosis was based on the results of operation and pathology. The inclusion criteria were as follows: (1) patients between 18 and 80 years; (2) patients with complete clinical data and confirmed breast lesions; and (3) all patients with single lesions received mammography, CTLM imaging, and postoperative pathological examination. The exclusion criteria were as follows: (1) had received breast lesions related treatment one month before examination; (2) had breast augmentation surgery with implants in the breast; (3) a history of allergic symptoms to light; (4) pregnant or nursing patients; and (5) incomplete clinical data, lack of mammography, CTLM imaging, and postoperative pathological examination. The final total included 225 patients. All were females, including 89 patients with malignant breast tumor, aged 24–79 years, with a mean age of 50.33 ± 10.58 years, and 136 patients with benign breast lesions, aged 31–70 years, with a mean age of 46.62 ± 6.98 years. The study was a retrospective analysis with no informed written consent from the patients. Before analysis, all records are anonymized and stripped of identity.

### 2.2. Instruments and Methods

(1) Mammography: the full digital mammography machine (Selenia Dimensions, Hologic, USA) was used for breast examination. The patient was placed in a standing position, and radiographs of both breasts were taken in the head and tail and in the external oblique position, with point compression and other views as appropriate. The main calculation of breast density, observation of calcification, and lesion location. (2) CTLM imaging: Imaging Diagnostic Systems of model 1020 CTLM is used for detection. The patient lies flat on the examination table in a prone position, fully exposing the examination area. A scan ring of an appropriate size is selected, and the laser source detector surrounds the area to be inspected. The section thickness is set to 2 mm by default, which can be adjusted according to the size of the patient's breast. If the breasts are too large, it is set to 4 mm. If the breasts are too small, it is set to 1 mm. After scanning, 3D image reconstruction is carried out using special software. Image interpretation is performed by radiologists with at least 5 years of working experience.

### 2.3. Observation Indexes

1. The results of the postoperative pathological examination of 225 patients were recorded and the image characteristics of CTLM were analyzed
2. The patients were divided into benign tumor group and malignant tumor group. The differences of general clinical data and image features of CTLM imaging were compared between the two groups
3. Compared with the pathological results, the detection rate of benign and malignant tumors and abnormal lesions on mammography and CTLM were analyzed, and the sensitivity, specificity, positive predictive value (PPV), and negative predictive value (NPV) of the two methods were calculated and also comparative diagnostic efficacy was carried out
4. To explore whether the classification of different clinical indicators can affect the detection rate of abnormal lesions by CTLM imaging

### 2.4. Statistical Analysis

SPSS 25.0 statistical software package was used for data analysis. Quantitative parameters in this paper were expressed in the form of the mean ± standard deviation (*X* ± *S*). Intergroup analysis was performed using the independent sample *t*-test. The images were drawn using the GradPad Prism 7.0 software package. Enumeration data were presented in the form of (%), and differences between groups were compared using *χ*^2^ analysis. The significance level was 0.05.

The article "Consistency Analysis of CTLM Imaging and Mammography in the Diagnosis of Breast Tumor Lesions" was retracted in 2023. Reasons: signs of a paper mill; suspected computer-generated content; unreliable results or conclusions; lack of ethics approval or compliance.

## 3. Results

### 3.1. Pathological Results and General Clinical Data of Enrolled Patients

According to the inclusion criteria and exclusion criteria established according to the purpose of the study, a total of 225 patients were included as research objects. Pathological results showed that 136 cases (60.44%) of breast tumors were benign tumors. There were 74 (32.89%) fibroadenomas, 38 (16.59%) adenopathy, 19 (8.44%) intraductal papilloma, 2 (0.89%) chronic inflammation, and 3 (1.33%) lobulated tumors of the breast. 89 patients (39.56%) were found with malignant tumors, including 40 (17.78%) with invasive lobular carcinoma, 36 (16%) with invasive ductal carcinoma, 2 (0.89%) with invasive ductal lobular carcinoma, 3 (1.33%) with ductal carcinoma in situ, 2(0.89%) with lobular carcinoma in situ, 2(0.89%) with microinfiltrating carcinoma, and 4 (1.78%) with other tumors. The patients were divided into the benign tumor group and the malignant tumor group. There were significant differences in age, BMI, and menstrual status between the two groups (*P* < 0.05). There was no significant difference between groups with hormone use history and family history of breast lesions (*P* > 0.05). The results are in Table 1 and 2.

### 3.2. CTLM Image Features of Normal and Abnormal Breast

In CTLM imaging, blood hemoglobin is the body's natural contrast agent. By comparing the image features of normal and abnormal blood vessels, the image features of attenuation signal of abnormal blood vessels were summarized in Figure 1. In CTLM imaging, the normal vascular signal structure of the breast was mainly manifested as banded, branched, and stellate structures. The branching or stellate structures are usually formed by intersecting veins. In this study, the normal CTLM images of blood vessels are thicker near the chest wall and converge toward the nipple, and gradually become thinner when converging, and when converging in the areola region, a flat round high signal intensity region (or bright region) is formed. The blood distribution of normal glandular lobules in the coronal image is shown as multiple cone-shaped regions with tips pointing to the center, showing a “spoke-like” distribution. The image can be observed layer by layer on the coronal image, and this image representation is continuously changing. Abnormal vascular morphology in coronal images is usually manifested as round or oval bright signal or high signal intensity areas, and is often accompanied by a layer-by-layer interruption of the “hub-like distribution” of the glandular lobules. In the 3D reconstruction images, the abnormal angiogenic areas were mostly irregular nonbanded structures, manifested as slab structure, spindle structure, spherical structure, diverticulum structure, inverted conical structure, rings structure, branched structure and dumbbell structure, and were shown in MIP mode, but rarely appeared in FTB mode. The angiogenic area of malignant tumors is also shown as an isolated area of high signal intensity, which is less associated with the surrounding areas of low signal intensity.

The article "Consistency Analysis of CTLM Imaging and Mammography in the Diagnosis of Breast Tumor Lesions" was retracted in 2023. Reasons: signs of a paper mill; suspected computer-generated content; unreliable results or conclusions; lack of ethics approval or compliance.

### 3.3. Comparison of CTLM Image Features of Benign and Malignant Breast Tumor

Benign and malignant tumors have different CTLM image characteristics. The classification and summary of the image features of benign and malignant tumors are helpful to the diagnosis of benign and malignant breast tumors. Compared with CTLM images of normal patients, the abnormal focus image signal area has a significant bright area, interrupting the regular distribution, color for bright white or yellow-green. The results of the 3D reconstruction showed that the shape of the abnormal area was more like a slab structure, a spindle structure, a spherical structure, and a diverticulum structure. The areas of malignant lesions were bright white (*P* < 0.001), and the margins with surrounding normal tissue were irregular (*P* < 0.001). The laser signal attenuation was obvious (*P* < 0.001), and the probability of 3D reconstruction shapes resembling slab structure, branch structure, ring structure, and dumbbell structure is higher than that of benign tumor lesions (*P* < 0.001). The high-intensity signal areas of benign lesions were yellow-green (*P* < 0.001), and the margins with surrounding normal tissue were regular (*P* < 0.001). The laser signal attenuation was moderate (*P* < 0.001), and the probability of the 3D reconstruction structure being spindle structure, spherical structure, and diverticulum structure is higher than that of the malignant tumor focus (*P* < 0.001). The results are in Table 3.

### 3.4. Consistency Analysis between CTLM Imaging and Pathological Examination

225 cases of patients with mammography and CTLM imaging, according to the image characteristics of the two detection methods, for the diagnosis of patients with lesions. Mammography diagnosis of breast showed that 101 cases were malignant (75 cases were pathologically malignant, 26 cases were benign), 69 cases were benign (8 cases were pathologically malignant and 61 cases were benign), and 55 cases were undetected (6 cases were pathologically malignant and 49 cases were benign). The total detection rate of breast tumors by mammography is 75.5% (170/225), and the detection rate of breast malignant tumors is higher than that of breast benign tumors, with a benign detection rate of 63.97% (87/136) and a malignant detection rate of 93.26% (83/89). CTLM imaging diagnosed 105 cases as malignant (78 cases as pathological malignant and 27 cases as benign), 85 cases as benign (7 cases as pathological malignant and 78 cases as benign), and 35 cases as undetected (4 cases as pathological malignant and 31 cases as benign). The total detection rate of CTLM imaging for breast tumors was 84.44% (190/225), and the detection rate for breast malignant tumors was higher than that for breast benign tumors, with the benign detection rate of 77.20% (105/136) and the malignant detection rate of 95.50% (85/89). The sensitivity, specificity, PPV, and NPV of the two assays were calculated. The specificity and diagnostic coincidence rate of CTLM imaging were higher than those of mammography (*P* < 0.05). The results are in Table 4, Table 5, and Figure 2.

The article "Consistency Analysis of CTLM Imaging and Mammography in the Diagnosis of Breast Tumor Lesions" was retracted in 2023. Reasons: signs of a paper mill; suspected computer-generated content; unreliable results or conclusions; lack of ethics approval or compliance.

### 3.5. Influences of Different Clinical Indicators on the Detection Rate of CTLM Lesions

Different clinical indicators may affect the diagnostic results of CTLM imaging. 89 patients were classified, and the detection rates of CTLM imaging in different breast densities, tumor sizes, estrogen receptor (ER), progesterone receptor (PR), and human epidermal growth factor receptor -2 (HER2) expression were compared. The results showed that there was no statistical difference in the detection rate of CTLM imaging in the classification of different breast densities, tumor focus sizes, ER, PR, HER2, and other markers (*P* > 0.05). The results are in Table 6.

## 4. Discussion

Breast cancer is the most common cancer in women, with a higher mortality rate. For breast cancer, the prevention and treatment are mainly regular screening, early detection of abnormal lesions, according to the type of lesions and tumor size to formulate the corresponding treatment plan [11]. The early detection of abnormal lesions is mainly due to regular physical examination, which mainly includes clinical palpation and routine imaging examinations such as mammography, MRI, and B-ultrasound [12, 13]^.^ Accurate diagnosis of lesion types and measurement of primary tumor size can help doctors make appropriate treatment plans before operation, and accurately evaluate the progress of lesions and the efficacy of neoadjuvant therapy in the course of treatment.

In this study, 225 patients with breast tumors were analyzed retrospectively. CTLM imaging and mammography were performed in all patients. Mammography was used as the routine imaging control, and postoperative pathological examination was taken as the gold standard. The CTLM image characteristics of breast lesions by CTLM imaging were analyzed, and the consistency of CTLM imaging in the diagnosis of breast lesions was calculated. The image characteristics of CTLM imaging were analyzed, the differences of image features between benign and malignant breast tumors were compared, and the common points of image identification were summarized. Use different clinical indicators to classify patients and explore the impact of different clinical indicators on the detection rate of CTLM imaging. To further discuss the clinical value of CTLM imaging in breast cancer.

The article "Consistency Analysis of CTLM Imaging and Mammography in the Diagnosis of Breast Tumor Lesions" was retracted in 2023. Reasons: signs of a paper mill; suspected computer-generated content; unreliable results or conclusions; lack of ethics approval or compliance.

Mammography is a common method for screening breast cancer. Mammography includes two positions: head-tail position and internal and external oblique positions. Breast density will affect the radiographic results. On mammograms, low-density tissue appears to be translucent, a dark gray shadow close to a black background. When the patient has a dense breast, the breast tissue density increases, and the film looks whiter on a gray background. The tumor in the focal area is also composed of dense tissue, so the film will also show white [14]. As a result, the tissue in the focus area of dense breast patients cannot form an obvious contrast with the surrounding normal tissues, which leads to measurement errors [15]. In this study, we compared the tumor detection rate of CTLM imaging in patients with dense breast and fatty breast. The results showed that there was no statistical difference in the detection rate between the two groups. It shows that the breast density of the patient will not interfere with the diagnostic structure of CTLM imaging.

If the tumor in abnormal breast lesions is to grow into a mass larger than 1 mm^3^, new blood vessels need to be generated [16]. Neovascularization in tumor cannot only nourish the surrounding tumor tissues [17], but also secrete various factors to induce the proliferation and migration of tumor cells. Therefore, it is of great clinical significance to monitor abnormal angiogenesis in the lesion. CTLM imaging is an optical imaging technology characterized by noninvasive and nonradiation. In CTLM imaging, there is no need to inject additional contrast agents, and deoxyhemoglobin in blood can be used as the natural contrast agent of the human body. Therefore, the high-density deoxyhemoglobin region can be quickly found. Three-dimensional image reconstruction is carried out on the image of this area, and the image features are analyzed. By analyzing the abnormal hemoglobin generation in the diseased area, it is judged whether there is abnormal angiogenesis in this area.

The article "Consistency Analysis of CTLM Imaging and Mammography in the Diagnosis of Breast Tumor Lesions" was retracted in 2023. Reasons: signs of a paper mill; suspected computer-generated content; unreliable results or conclusions; lack of ethics approval or compliance.

In this study, according to the results of postoperative pathological examination, among 225 breast patients, 136 cases were benign tumors and 89 cases were malignant tumors. Analysis of CTLM imaging results showed that 190 patients (84.44%) were abnormal, and the detection rate of benign breast lesions was 77.20%, and the detection rate of malignant breast lesions was 95.50%. The consistency between CTLM imaging and postoperative pathological examination was calculated. The results showed that the sensitivity, specificity, NPV, PPV, and diagnostic coincidence rate of CTLM imaging were 87.64%, 57.35%, 91.76%, 74.29%, and 69.33%, respectively. The consistency of CTLM imaging in diagnosis and pathological examination of breast tumors is higher than that of mammograms, which is considered to be related to the high proportion of heterogeneous dense breast and extremely dense breast in the population of this study.

CTLM imaging is mainly aimed at tumor neovascularization in the focus area. The vascular structure of benign and malignant lesions is different [18], partly influenced by tumor angiogenesis factors. Tumor cells in malignant lesions grow faster and need a more abundant blood supply. Therefore, the secretion of angiogenic factors in malignant lesions increases, which increases the speed of vascular growth. There are many new blood vessels, but the basic structure of blood vessels is incomplete, lacking vascular endothelial cells, smooth muscle cells, and nerve endings [19]. The systolic and diastolic function of malignant blood vessels is lost, the wall of blood vessels is thin, and the diameter of blood vessels is increased. When CTLM imaging is performed, there are areas with high local hemoglobin content, which appear as local bright white on the image, destroying the original regular radial distribution. Irregular edges of lesions and surrounding normal tissues, obvious attenuation of laser signals, and the shape of 3D reconstruction similar to plate-like structures are also interpreted as signs of malignant lesions. Image features are consistent with those reported by researchers such as Qi [20]. When CTLM imaging is performed on benign and malignant lesions, the two lesions will show different image features. In this study, the detection rate of malignant tumors by CTLM imaging was higher than that of benign tumors. Nevertheless, since CTLM is a functional examination, there are some limitations in accurately locating the lesions.

In conclusion, CTLM can reflect the information of breast cancer neovascularization to some extent, and the results of image identification are consistent with the results of pathological examination. CTLM imaging can be used as an auxiliary examination in the diagnosis of breast cancer lesions with a certain clinical value.

The article "Consistency Analysis of CTLM Imaging and Mammography in the Diagnosis of Breast Tumor Lesions" was retracted in 2023. Reasons: signs of a paper mill; suspected computer-generated content; unreliable results or conclusions; lack of ethics approval or compliance.

## Figures and Tables

**Figure 1:** CTLM image features of normal and abnormal breast (A–C) normal vascular signal structure of the breast: banded structure (a), branched structure (b), and stellate structure (c); (d) Coronal plane normal glandular lobules “spokes” distribution; (e) Oval-shaped bright signal area on the coronal plane of CTLM, showing abnormal angiogenesis and “spoke-like” distribution interruption; F–I : the abnormal vascular signal structures in the breast are indicated by the red arrow: ring structure (f), spindle structure (g), diverticulum structure (h), and plate structure (i).

**Figure 2:** Comparison of diagnostic efficacy between mammography and CTLM in 225 breast patients.

**Table 1:** Pathological results of 225 patients with breast tumor.

Benign and malignant	Category	Ratio of patients N (%)
Benign tumour, *n* = 136 (60.44%)	Fibroadenoma	74 (32.89)
	Adenopathy	38 (16.89)
	Intraductal papilloma	19 (8.44)
	Chronic inflammation	2 (0.89)
	Lobulated tumor of the breast	3 (1.33)
Malignant tumor, *n* = 89 (39.56%)	Invasive lobular carcinoma	40 (17.78)
	Invasive ductal carcinoma	36 (16.00)
	Invasive ductal lobular carcinoma	2 (0.89)
	Ductal carcinoma in situ	3 (1.33)
	Lobular carcinoma in situ	2 (0.89)
	Microinfiltrating carcinoma	2 (0.89)
	Others	4 (1.78)
Total		225 (100)

**Table 2:** Comparison of general clinical features of 225 patients with breast tumor.

Classification	Benign tumor (*n* = 136)	Malignant tumors (*n* = 89)	*P Value*
Age (years)	46.62 ± 6.98	50.33 ± 10.58	0.001
BMI (kg/m^2^)	23.26 ± 3.51	24.10 ± 3.13	0.021
*Menstrual status n* (%)			
Premenopausal	96 (70.59)	41 (46.07)	0.000
Postmenopausal	40 (29.41)	48 (53.93)	
Hormone use, *n* (%)	1 (0.74)	2 (2.25)	0.397
History of benign breast lesions, *n* (%)	8 (5.88)	4 (4.49)	0.578
Family history of breast malignancy, *n* (%)	22 (16.18)	18 (20.22)	0.740

*Note.* BMI is body mass index.

**Table 3:** Comparison of CTLM image features of benign and malignant breast tumors.

Image characteristics	Benign tumour (*n* = 105)	Malignant tumor (*n* = 85)	*P value*
*Region color*			
Bright white	49 (46.67)	72 (84.71)	0.000
Green and yellow	56 (53.33)	13 (15.29)	
*Focal edge*			
Regular	34 (32.38)	7 (8.24)	0.000
Irregular	71 (67.62)	78 (91.76)	
*Laser signal attenuation*			
Weak	8 (7.62)	2 (2.35)	0.000
Medium	76 (72.38)	24 (28.24)	
Obvious	21 (20.00)	59 (69.41)	
*3D structure*			
Slab structure	13 (12.38)	29 (34.12)	0.000
Spindle structure	34 (32.38)	21 (24.71)	
The spherical structure	25 (23.81)	3 (3.53)	
Diverticulum structure	23 (21.90)	16 (18.82)	
Inverted conical structure	7 (6.67)	1 (1.18)	
Rings structure	1 (0.95)	6 (7.06)	
Branched structure	1 (0.95)	4 (4.71)	
Dumbbell structure	1 (0.95)	5 (5.88)	

The article "Consistency Analysis of CTLM Imaging and Mammography in the Diagnosis of Breast Tumor Lesions" was retracted in 2023. Reasons: signs of a paper mill; suspected computer-generated content; unreliable results or conclusions; lack of ethics approval or compliance.

**Table 4:** Comparison of the detection rate of benign and malignant lesions by mammography and CTLM imaging.

Inspection method		Pathological result		Total	*P*
		Benign	Malignant		
Mammography	Malignant	26	75	101	0.000
	Benign	61	8	69	
	Not detected	49	6	55	
	Total	136	89	225	

CTLM	Malignant	27	78	105	0.000
	Benign	78	7	85	
	Not detected	31	4	35	
	Total	136	89	225	

**Table 5:** Comparison of diagnostic performance of mammography and CTLM imaging in 225 breast patients.

	Breast X-ray	CTLM imaging	*P*
Sensitivity (%)	84.26 (75/89)	87.64 (78/89)	0.518
Specificity (%)	44.85 (61/136)	57.35 (78/136)	0.039
NPV (%)	88.41 (61/69)	91.76 (78/85)	0.484
PPV (%)	74.26 (75/101)	74.29 (78/105)	0.622
Coincidence rate	60.44 (136/225)	69.33 (156/225)	0.048

*Note.* NPV is negative predictive value, and PPV is positive predictive value.

**Table 6:** Influence of different clinical indicators on the detection rate by CTLM in 89 breast cancer.

Index	Type	CTLM imaging		
		Detection *n* (%)	Not detected *n* (%)	*P*
Breast density	Dense type	69 (81.2)	4 (100)	0.202
	Lard type	16 (18.8)	0 (0.0)	
Tumor size	≤2 cm	47 (55.3)	2 (50.0)	0.659
	2–5 cm	31 (36.5)	2 (50.0)	
	>5 cm	7 (8.2)	0 (0.0)	
ER	+	70 (82.4)	2 (50.0)	0.153
	-	15 (17.6)	2 (50.0)	
PR	+	46 (54.1)	3 (75.0)	0.399
	-	39 (45.9)	1 (25.0)	
HER2	+	34 (40.0)	2 (50.0)	0.693
	-	51 (0.0)	2 (50.0)	
Ki67	<14	7 (8.2)	0 (0.0)	0.413
	≥14	78 (91.8)	4 (100.0)	

## Data Availability

All the data including statistical analysis has been presented in this paper.
